# Gabor Dictionary of Sparse Image Patches Selected in Prior Boundaries for 3D Liver Segmentation in CT Images

**DOI:** 10.1155/2021/5552864

**Published:** 2021-12-09

**Authors:** Xuehu Wang, Zhiling Zhang, Kunlun Wu, Xiaoping Yin, Haifeng Guo

**Affiliations:** ^1^College of Electronic and Information Engineering, Hebei University, Baoding 071002, China; ^2^Research Center of Machine Vision Engineering and Technology of Hebei Province, Baoding 071002, China; ^3^Key Laboratory of Digital Medical Engineering of Hebei Province, Baoding 071002, China; ^4^Hebei Research Institute of Construction and Geotechnical Investigation Co.,Ltd., Shijiazhuang, Hebei, China; ^5^Affiliated Hospital of Hebei University, Baoding 071000, China

## Abstract

The gray contrast between the liver and other soft tissues is low, and the boundary is not obvious. As a result, it is still a challenging task to accurately segment the liver from CT images. In recent years, methods of machine learning have become a research hotspot in the field of medical image segmentation because they can effectively use the “gold standard” personalized features of the liver from different data. However, machine learning usually requires a large number of data samples to train the model and improve the accuracy of medical image segmentation. This paper proposed a method for liver segmentation based on the Gabor dictionary of sparse image blocks with prior boundaries. This method reduced the number of samples by selecting the test sample set within the initial boundary area of the liver. The Gabor feature was extracted and the query dictionary was created, and the sparse coefficient was calculated to obtain the boundary information of the liver. By optimizing the reconstruction error and filling holes, a smooth liver boundary was obtained. The proposed method was tested on the MICCAI 2007 dataset and ISBI2017 dataset, and five measures were used to evaluate the results. The proposed method was compared with methods for liver segmentation proposed in recent years. The experimental results show that this method can improve the accuracy of liver segmentation and effectively repair the discontinuity and local overlap of segmentation results.

## 1. Introduction

Liver cancer is one of the most common cancers in the world and one of the most common causes of cancer death [1, 2]. Medical imaging is considered to be an important technology to help doctors assess diseases, optimize prevention, and control measures. In recent years, computed tomography (CT) has become widely used in clinical medical diagnosis and treatment due to its high spatial resolution and fast imaging speed [3–5]. At present, many studies focus on how to improve the accuracy and efficiency of liver segmentation, but there are still many problems to be solved, such as the complex shape of the liver, low contrast between the liver and adjacent organs, and no obvious boundary.

Against such a backdrop, the method based on machine learning has developed rapidly and become a research hotspot in recent years. Researchers have proposed a large number of liver segmentation methods, such as region growth, graph cut algorithm, level set, active contour, statistical shape model, and clustering [6–11]. The method based on image segmentation is simple to operate, but the segmentation effect is unstable and easily affected by the contrast between the liver and surrounding organs. The segmentation method based on the model has stable performance but requires multiple annotation data and high requirements for registration. The clustering method does not need image annotation and is an unsupervised learning method. Deep learning is a branch of machine learning algorithms. It can learn rules from a large number of labeled datasets for liver training, determine the parameters of the segmentation model, automatically extract deep features of the liver, and segment the liver, thereby reducing the impact of human factors on the segmentation results [12, 13]. However, every deep learning model built is for specific data, resulting in poor versatility. Both of these methods require a large amount of data, which reduces the efficiency of segmentation. How to reach a balance between the amount of sample data and the segmentation accuracy has become a major difficulty in medical image segmentation [14]. To improve the efficiency of machine learning-based algorithms, technologies such as the K-SVD (Singular Value Decomposition) algorithm, sparse code, and inquiry dictionaries have been widely applied. Zhang et al. [15] proposed a sparse optimization model based on prior knowledge that segmented the liver surface into many subregions and used the K-SVD algorithm to establish the shape information dictionary of the liver, thereby constraining the deformation model to approach the liver boundary with sparse it. Liao et al. [16] replaced voxel information with features of local image patches and constructed a sparse dictionary model for liver segmentation, which improved the segmentation accuracy of the low-contrast regions to a certain extent. Wang et al. [17] used the best sparse combination of shapes in the sample database to represent the liver shape without any assumptions regarding its parameter distribution. This method can obtain the prior shape of the liver accurately and rapidly from a large number of samples. Shi et al. [18] proposed a prior shape model based on the low-rank sparse decomposition, which reduced the limitations on the application of the PCA dimension reduction for existing statistical shape models. Xu et al. [19] built an inquiry dictionary for the target region in the training image with this method, divided the target image into image patches of the same size to construct a test set, and then defined the target boundary according to the matching degree of the test set and the inquiry dictionary. Wang et al. [20], by using the sparse representation of high-dimensional medical structures based on tensors, not only successfully retained the spatial structure inherent in high-dimensional medical data but also captured the time information in multiphase medical images.

Although great progress has been made in algorithms for liver segmentation based on sparse code, previous research has shown [11] that the similarity of judgments over small image patches would seriously affect the accuracy of segmentation, and most existing algorithms, using a grayscale dictionary to compare the similarity of images, will have lower matching accuracy. In addition, the segmentation results of existing methods present different degrees of voids and overlaps, which in turn affect the segmentation accuracy.

There are two novelties in this method: (1) by extracting Gabor features, the boundary information of the liver can be better extracted, and a sparse coding method is adopted to reduce the number of training samples and remove redundant information; (2) the segmentation results were effectively repaired by cavity filling, and the redundant boundary points were removed, so as to obtain a smooth liver boundary.

## 2. Methods

### 2.1. The Overall Process of the Proposed Algorithm

The flow chart of the proposed approach is illustrated in Figure 1. First, the abdominal image with the “gold standard” was registered with the abdominal image to be segmented through the registration technology, and Gabor feature extraction was performed on the registered image, and the “gold standard” after the registration is defined as the initial boundary of the liver. Second, select N image blocks of the same size as the training set on the liver boundary of the Gabor feature image with the “gold standard” and then use the K-SVD algorithm to train the query dictionary and the corresponding sparse coding. Third, select all voxel points in the ten neighborhoods with each point on the initial boundary of the liver as the center, and select the image blocks with the same size as the training set as the boundary point with each voxel point in the neighborhood as the center test set. Fourth, use the trained query dictionary and the test set (Orthogonal Matching Pursuit, OMP) algorithm to calculate the sparse coding corresponding to the test set. Finally, an operation for hole filling is performed on the obtained liver boundary to obtain the final segmentation result.

### 2.2. Liver Region Registration

To register the gold standard image and image to be segmented, this paper, after referring to previous laboratory studies [21], selects the corresponding marked points in the training image and the target image, determines the deformation field according to the matching relationship between these points, and applies the deformation field to the gold standard image. In this way, the approximate position and contour of the liver in the target image are obtained. The registration flow chart is shown in Figure 2.

If the entire CT image is used to register the training image and the target image, the liver region will be affected by other similar density soft tissues, resulting in lower registration accuracy [22]. To solve this problem, this paper manually selected five sets of feature point pairs in the training image and the target image, establishes the deformation relationship between the feature points, uses the B-spline interpolation method to calculate the overall deformation relation *V*_*o*_ ship of the liver, and thereby constructs the deformation field between the volume data. The method of calculating the initial boundary of the liver in the test image is as follows.

The training image is defined as *V*_*o*_. Its corresponding gold standard liver image is *V*_*s*_, and the target image is *V*_*u*−*s*_. In this light, the registration calculation process of and *V*_*u*−*s*_ is as follows:

(1) $$\begin{array}{c} s_{\text{opt}}=\arg\;\min\left(\text{Sim}\left(V_{u-s},V_{o}\circ s_{i},s\right)+{\left\|s\right\|}^{2}\right). \end{array}$$

In this process, *s*_opt_ is the optimal deformation field, *s*_*i*_ is the original deformation field obtained via the registration of the marked points, Sim(*∗*) refers to similarity measure, ‖*∗*‖ refers to the regularized constraint of the deformation field, and “∘” indicates the application of the deformation field to the abdominal volume data. The optimal deformation field *s*_opt_ is applied to the gold standard image *I*_*s*_ to obtain the approximate location and contour of the liver in the target image *I*_*i*−*s*_. The calculation process is as follows:

(2) $$\begin{array}{c} I_{i-s}=I_{s}\circ s_{\text{opt}}. \end{array}$$

### 2.3. Training Dictionary

So far, researchers have proposed various different sparse dictionaries, i.e., the wavelet dictionary, the local cosine dictionary, the Anisotropic Refinement Gaussian (AR-Gaussian) multicomponent dictionary, etc. [23–26]. Among all these dictionaries, the separability and isotropy of wavelet atoms seriously affect the ability of the dictionary to describe the boundary structure of images. The local cosine dictionary, though it can effectively match the texture structure of images, cannot effectively demonstrate the edge contour structure of images. If the Gaussian function and second derivative are used as the atom generating function, the edge structure of images can be matched effectively, but the dictionary contains a huge number of atoms, which increases the complexity of the sparse decomposition. For specific image modes, effective image representation methods must be selected. Similarly, as for liver CT images, Gabor feature images are a good choice for building dictionaries. Therefore, this paper established a Gabor dictionary of images (for information on the extraction of the Gabor features of images, please refer to previous research results [11, 27]). Ten neighborhood image patches are selected as the training set of the Gabor feature dictionary from the liver boundary in an abdominal Gabor image with the “gold standard” liver (as shown in Figure 3).

In this paper, we adopted the K-SVD algorithm [28] to train the Gabor feature dictionary on the liver boundary. The algorithm is a circulatory learning process. Given a training set *Y*_training_ and by defining an overcomplete dictionary $D=\left\{{\overset{⟶}{d}}_{m1},{\overset{⟶}{d}}_{m2},\ldots ,{\overset{⟶}{d}}_{mt}\right\}\in R^{m\times t}$ in which *m* is the number of rows of vector ${\overset{⟶}{d}}_{m1}$, *t* is the number of atoms of the dictionary, *m* < *t*, where *X*_training_ is the sparse coefficient of the dictionary, and *T*_0_ is the sparseness; the signal can be then represented by a sparse linear dictionary atom, which can be shown as follows:

(3) $$\begin{array}{c} \langle D,X_{\text{training}}\rangle =\underset{D,X_{\text{training}}}{\min}\left\{{\left\|Y_{\text{training}}-DX_{\text{training}}\right\|}_{F}^{2}\right\}\text{s.t.}\;\forall i,\left\|x_{i}\right\|\leq T_{0}. \end{array}$$

In this process, *D* has been normalized via the following formula:

(4) $$\begin{array}{c} D=\left\{{\overset{⟶}{d}}_{m1},\ldots ,{\overset{⟶}{d}}_{mt}\right\}\\ =\left\{\frac{{\overset{⟶}{d}}_{m1}}{{\left\|{\overset{⟶}{d}}_{m1}\right\|}_{2}},\ldots ,\frac{{\overset{⟶}{d}}_{mt}}{{\left\|{\overset{⟶}{d}}_{mt}\right\|}_{2}}\right\}. \end{array}$$

Such an optimization problem can be solved in the following two steps.

#### 2.3.1. Sparse Coding

At this stage, we assume that dictionary *D* is fixed and take the optimization problem in formula (3) as a process of finding optimal sparse coefficients *X*_training_ in matrix *X*. Then, the above formula can be modified as follows:

(5) $$\begin{array}{c} {\left\|Y_{\text{training}}-DX_{\text{training}}\right\|}_{F}^{2}=\sum_{i=1}^{N}{\left\|y_{i}-Dx_{i}\right\|}_{2}^{2}. \end{array}$$

Therefore, the optimization problem can be modified as follows:

(6) $$\begin{array}{c} \langle X_{\text{training}}\rangle =\underset{D,X_{\text{training}}}{\min}\left\{\sum_{i=1}^{N}{\left\|y_{i}-Dx_{i}\right\|}_{2}^{2}\right\}\;\text{s.t.}\;{\left\|x_{i}\right\|}_{0}\leq T_{0}. \end{array}$$

In the formula, *i*=1,2,…, *N*. *x*_*i*_ and *y*_*i*_ are the coordinates of the graph. If *T*_0_ is small enough, the problem can be solved with the OMP [29] algorithm.

#### 2.3.2. Dictionary Update

Assuming that coefficient *X*_training_ and dictionary *D* are both fixed, the kth column ${\overset{⟶}{d}}_{k}$ of the dictionary shall be updated while all the columns in the sparse matrix *X* are multiplied by the kth row in ${\overset{⟶}{d}}_{k}$ that shall be recorded as *x*_*T*_^*k*^. In this light, target function (3) can be rewritten as follows:

(7) $$\begin{array}{c} \langle D\rangle ={\left\|y_{i}-Dx_{i}\right\|}_{F}^{2}={\left\|Y_{\text{training}}-\sum_{j=1}^{K}{\overset{⟶}{d}}_{j}x_{T}^{j}\right\|}_{F}^{2}={\left\|\left(Y_{\text{training}}-\sum_{j\neq k}{\overset{⟶}{d}}_{j}x_{T}^{j}\right)-{\overset{⟶}{d}}_{j}x_{T}^{j}\right\|}_{F}^{2}={\left\|E_{k}-{\overset{⟶}{d}}_{j}x_{T}^{j}\right\|}_{F}^{2}. \end{array}$$

We decompose *DX*_training_ into the sum of matrix *K* (rank: 1) and assume that *K* − 1 is fixed while the remaining one column is the *k*th column to be updated, representing the error rate relative to the original training set after removing atoms in the *E*_*k*_ column. Then, we only keep nonzero elements for *E*_*k*_ and *x*_*T*_^*k*^ and update ${\overset{⟶}{d}}_{k}$ with the SVD algorithm.

#### 2.3.3. Image Reconstruction

After obtaining the inquiry dictionary *D* and corresponding sparse code *X*_training_ with the training samples, we select ten neighborhood points in the *x*, *y*, and *z* directions at the vertex of the initial liver boundary of the image to be segmented, which results in a total of 30 neighborhood points, and use these 30 neighborhood points as the center to select 30 test sample sets with the same size as the training sample set to form the test sample set. The sparse code corresponding to the test samples is calculated by using the trained inquiry dictionary. We calculate the reconstruction error of each group of samples through the test samples, the inquiry dictionary, and sparse coding. The formula is as follows:

(8) $$\begin{array}{c} L_{\text{patch}}=\min\left(Y_{\text{testing}}^{i}-D_{\text{gabor}}X_{\text{gabor}}\right),\;\left(i=1,2,\ldots ,1000\right). \end{array}$$

The image patch with the smallest reconstruction error is selected as the liver boundary patch to calculate the center of each boundary patch and it is used as the boundary point of the liver.

### 2.4. Void Filling

The algorithm proposed in this paper uses image patches as the dictionary sample set, and the liver boundary obtained may display discontinuity or even boundary overlaps. In this paper, the surface convex hull algorithm [29] and the void-filling algorithm [30] are introduced to realize the interpolation and completion of the discontinuous region on the liver boundary and thereby obtain a smooth and continuous liver surface. The detailed calculation process is as follows:

1. Input the liver segmentation result, and use the Scan-conversion algorithm to perform octree decomposition, decomposing the segmentation result into a more refined subspace.
2. Suspend the octree decomposition when the intersections between all the decomposition lines and the original model are all located on the leaves of the octree.
3. Mark the boundary with intersections as an “intersecting edge.”
4. Select a vertex from the original model and mark it as “0.” Extend it along the boundary of the octree, and when it passes the “intersecting edge” once, the label will change to “1.” The rest may be deduced by analogy. Every time the intersecting boundary is passed, the label would change once, which would continue until the entire octree traversal ends.
5. Reconstruct the vertexes that only contain “0”s and “1”s accurately with the Dual Contouring algorithm to obtain the model after void filling.

## 3. Experiments

### 3.1. Datasets

This article tested our method on the MICCAI 2007 (https://www.sliver07.org/index.php) dataset and the ISBI2017 dataset and validated it on image data from the Affiliated Hospital of Hebei University. The MICCAI 2007 train dataset contains 20 contrast-enhanced CT volumes with standard segmentation, all of which have a pixel spacing of 0.55 to 0.8 mm, and a slice spacing of 1 to 3 mm, without any overlap between the slices. The ISBI2017 dataset contained 131 and 70 contrast-enhanced three-dimensional abdominal CT scans, which were used for training and testing, respectively. The dataset was obtained from six different clinical sites through different scanners and protocols, with a large difference in planar resolution from 0.55 mm to 1.0 mm and slice spacing from 0.45 mm to 6.0 mm. The dataset of the hospital contains 100 contrast-enhanced CT volumes. The pixel spacing and slice thickness vary from 0.64 to 0.65 mm and 5.0 mm, respectively, with the in-plane resolution of pixels in all cases.

To validate the proposed method, experiments were conducted on a Windows 10 personal computer (PC) with an Intel i7-7700K CPU and Nvidia GPU RTX3090. The proposed algorithm was implemented in Python. The insight segmentation and registration toolkit ITK (https://www.itk.org/) and the visualization toolkit VTK (https://www.vtk.org/) were used for basic 3D image processing and 3D visualization of segmentation results, respectively.

### 3.2. Evaluation Measures

To further verify the segmentation accuracy of the algorithm, the experiment applies five evaluation criteria provided by MICCAI 2007 for evaluation, including the following: the Volumetric Overlap Error (VOE), the Relative Volume Difference (RVD), the Average Symmetric Surface Distance (ASSD), the Root Mean Square Symmetric Surface Distance (RMSSSD), and the Maximum Symmetric Surface Distance (MSSD). The smaller the values of the five evaluation criteria are, the better the performance is. The region the of segmentation result is defined as *A* while the “gold standard” region is *B*. *S*(*∗*) is the surface voxel of data “*∗*” and refers to any point on the surface voxel. *D*(*∗*) refers to the Euclidean distance. The calculation processes of the five kinds of accuracy are as follows (for reference).

(1) Volume overlap error
  (9) $$\begin{array}{c} \text{VOE}=100\cdot \left(1-\frac{\left(\left|A\cap B\right|\right)}{\left(\left|A\cup B\right|\right)}\right). \end{array}$$
(2) Relative volume error
  (10) $$\begin{array}{c} \text{RVD}=100\cdot \left(\frac{\left(\left|A\right|-\left|B\right|\right)}{\left|B\right|}\right). \end{array}$$
(3) Average symmetrical surface distance
  (11) $$\begin{array}{c} \text{ASSD}=\frac{\left(\sum_{S_{A}\in S\left(A\right)}D\left(S_{A},S\left(B\right)\right)+\sum_{S_{B}\in S\left(B\right)}D\left(S_{B},S\left(A\right)\right)\right)}{\left(\left|S\left(A\right)\right|+\left|S\left(B\right)\right|\right)}, \end{array}$$
where *D*(*v*, *S*(*A*))=min_*S*_*A*_∈*S*(*A*)_‖*v* − *S*_*A*_‖, and ‖*∗*‖ is the Euclidean distance.
(4) Root mean square symmetric surface distance
  (12) $$\begin{array}{c} \text{RMSSSD}=\frac{\sqrt{\left(\sum_{S_{A}\in S\left(A\right)}D^{2}\left(S_{A},S\left(B\right)\right)+\sum_{S_{B}\in S\left(B\right)}D^{2}\left(S_{B},S\left(A\right)\right)\right)}}{\sqrt{\left(\left|S\left(A\right)\right|+\left|S\left(B\right)\right|\right)}}. \end{array}$$
(5) Maximum symmetrical surface distance
  (13) $$\begin{array}{c} \text{MSSD}=\max\left\{\underset{S_{A}\in S\left(A\right)}{\max}D^{2}\left(S_{A},S\left(B\right)\right),\underset{S_{B}\in S\left(B\right)}{\max}D^{2}\left(S_{B},S\left(A\right)\right)\right\}. \end{array}$$

## 4. Results

Before selecting the test set, it is necessary to register the gold standard image with the target image and then use the registered gold standard image as the initial boundary of the liver to be segmented. Therefore, the accuracy of the registration result directly affects the accuracy of the initial boundary and the test set. This paper selected two sets of gold standard images for registration used the initial boundary after registration and the gold standard to calculate the spatial distance error and thereby used this to evaluate the registration accuracy (as shown in Figure 4).  Figure 4(a) is the training image, Figure 4(b) is the gold standard image of the liver relative to Figures 4(a) and 4(e) is the target image. Points marked with (1)∼(5) in Figures 4(a) and 4(e) are selected marked points, which are used to register Figures 4(a)to 4(e). Registered Figure 4(a) is deformed into Figure 4(c) while the gold standard Figure 4(b) is deformed into Figure 4(d) under the impact of the deformation field.  Figure 4(f) is the posture of the registered gold standard image of the liver in the target image, proving that the registration method constructed in this paper can register the gold standard image and the target image accurately and obtain a relatively precise initial liver boundary, which also provides possible conditions for the selection of the appropriate training set.

This paper only selects the test set in the neighborhood of the initial boundary of the liver, which can effectively improve the segmentation efficiency. To test the accuracy of the region selection, 12 sets of CT data are used as the source images to be registered, two pairs of CT data are randomly selected for registration, and the deformation field after registration is applied to the gold standard image (as shown in Figure 5). Figures 5(a)∼5(f) show the visualization effects of the six sets of registration results in the gold standard image. The red region is the liver region in the target image, and the green region is the deformed gold standard liver region (the initial contour of the liver to be segmented). According to the figure, the liver boundary error after registration is very small (less than 10 voxels on average), which proves the feasibility of the algorithm proposed in this paper.

Since Gabor features are symmetrical features, this paper chose an angle every 20° within the range of 0 to 180° to form 972 Gabor filters with 243 angles and 4 scales. The Gabor filter bank convolutes with each image patch in airspace, and each image patch can obtain 972 filter outputs—images with the size of the image patch (as shown in Figure 6). If it is used as a feature vector directly, the dimensionality of the feature space will be very large. In this light, this paper selected the grayscale average value to form a 24 × 1 column vector as the Gabor feature of the image patch.

Figure 7 shows how the image patch selection results of the dictionary are displayed in the slice. Figures 7 (A1)∼(A3), (B1)∼(B3), and (C1)∼(C3) display the effects of the constructed dictionary image patches on the cross section, sagittal plane, and coronal plane, respectively. As seen from the figure, this paper selected the image patch on the liver boundary as the training set to ensure that the training set contains information about the liver boundary and thereby make the inquiry dictionary able to effectively express the features of the liver boundary.

Figure 8 shows the liver segmentation result obtained with sparse code and the training dictionary. Figures 8 (A1)∼(A3) and (B1)∼(B3) are the cross-sectional, sagittal, and coronal planes of the liver segmentation results of the two sets of CT data, respectively. Figures 8 (a1)∼(a3) and (b1)∼(b3) are the locally amplified views of the images in the green boxes of Figures 8 (A1)∼(A3) and (B1)∼(B3), respectively. It can be seen from the figure that the liver boundary obtained through sparse coding and dictionary querying is an image voxel point set with common features. If the liver boundary in the target image is blurred, a large number of image patches in the selected test set will match the inquiry dictionary, generating a relatively large amount of redundant information. However, when the image patches in the test set fail to match the grayscale information and Gabor feature information in the inquiry dictionary, the application of sparse coding and dictionary querying only would lead to voids on the liver boundary. After partially amplifying Figures 8 (a1), (a2), and (b1), it can be observed that the voxel points obtained on the liver boundary have generated a lot of overlapping redundant information, which will generate multiple liver boundaries and lead to inaccurate segmentation. According to Figures 8 (a3), (b2), and (b3), the liver boundary obtained through sparse coding and dictionary querying has produced discontinuous voids, which could lead to discontinuous segmentation results. To tackle this problem, this paper constructed a void-filling method to compensate for the discontinuity of the segmentation results. The specific results are shown in Figure 9.

Figure 9 shows the segmentation results of a set of 3D liver CT data. As seen from Figure 9 (a1), since the local boundary of the liver is not clear, it is difficult to find image patches that could be well matched with the inquiry dictionary in the test set, which has generated a relatively large number of overlapping regions in the segmentation result obtained through dictionary querying and sparse coding. In contrast, as for the segmentation after void filling, the liver boundary becomes smooth and free of voids (as shown in Figure 9 (a2)). In Figures 9 (b2) and (c2), the grayscale contrast between the liver boundary and its adjacent tissue is quite small, generating redundant boundary points in various regions of the segmentation result after void filling, which has reduced the segmentation accuracy. On the contrary, redundant boundary points have been eliminated from the results after void filling, obtaining a smooth liver boundary and fully proving the feasibility of the algorithm proposed in this paper.

Figure 9 shows the segmentation results of a set of 3D liver CT data. The first line is the segmentation result obtained by dictionary query and sparse coding method; the second line is the segmentation result after hole filling; the third line is the comparison chart of the segmentation result of this method and the gold standard. The fourth row to the sixth row are the enlarged images corresponding to the blue boxes in the first row to the third row, respectively. It can be seen from the fourth row of Figure 9 that because the local boundary of the liver is not clear, it is difficult to find an image block that matches the query dictionary well in the test set. This makes it appear that there are more blank and overlapping areas when using only query dictionaries and sparse coding methods. In contrast, for the segmentation result after hole filling, the liver boundary becomes smooth and there are no holes (as shown in the fifth row in Figure 9). In the first and second images in the fourth row in Figure 9, the grayscale contrast between the liver boundary and its adjacent tissues is very small, so that the segmentation results that have not undergone hole filling processing have redundant boundary points in multiple regions, which affects the accuracy of segmentation, and the result of hole filling effectively removes the redundant boundary points and obtains a smooth liver boundary, which fully proves the effectiveness of the algorithm in this paper.

Figure 10 shows five sets of randomly selected CT data and their liver segmentation results. The first to third columns in Figure 10 show the cross-sections, sagittal planes, and coronal planes of the segmentation results of original CT images. The red line in the figure represents the gold standard image of the liver manually segmented by experts, while the green line represents the liver segmentation result obtained with the algorithm proposed in this paper. According to the result shown in Figure 10, the boundary of the segmentation result is very consistent with the real boundary of the liver. The blurred liver boundary is also soundly segmented, which proves the efficiency of the Gabor dictionary in the algorithm and demonstrates the accuracy of selecting the test set on the initial boundary of the liver after registration. As can be seen from the third column in Figure 10 that the algorithm proposed in this paper can accurately segment the sharp corners and depression regions of the liver, which effectively proves that the inquiry dictionary established by this method can accurately represent the boundary features of the liver, and it can also soundly match the boundary features of sharp corners and depressed regions. In addition, the void-filling method has effectively repaired the void and redundant information of the segmentation result, obtained a smooth liver boundary, and improved the segmentation accuracy.

Figure 11 is a three-dimensional display comparison diagram of the liver segmentation results of five groups of randomly selected CT data. The second and third rows of Figure 11, respectively, show the liver segmentation results of the same CT before and after hole filling. The first and last rows of the figure show the partially enlarged images corresponding to the blue boxes in the second and third rows. As can be seen from the second row of the figure, the segmentation result before filling the holes has holes and the surface is not smooth. However, the segmentation results of the third row of Figure 11 after filling the holes are very smooth, and the grid information is continuous.

For the MICCAI 2007 dataset, Table 1 presents the results of the evaluation for segmentation accuracy of the proposed algorithm using five randomly selected CT data sets. The mean values of VOE, RVD, ASSD, RMSSSD, and MSSD after liver segmentation of the five groups of CT data by this algorithm were 4.7 ± 0.4%, 1.6 ± 0.7%, 0.8 ± 0.3 mm, 1.3 ± 0.5 mm, and 12.7 ± 5.1 mm, respectively. As can be seen from the values of ASSD and RMSSSD in the table, the construction of the liver surface void-filling algorithm in this algorithm makes the segmentation results have a high smoothness, which can basically make the surface of the segmentation results consistent with the surface of the gold standard liver. The total runtime was 25.43 s on average.

Table 2 lists the comparison results of the segmentation error between the method proposed in this paper and the six methods in the MICCAI2007. The methods of [9, 11, 33] are semiautomatic segmentation algorithms. The methods applied in [34], reference [31, 32] are automatic segmentation algorithms. Compared with the six algorithms in the references, through the dictionary established that can accurately represent the boundary features of the liver, the void-filling method has effectively obtained a smooth liver boundary and improved the segmentation accuracy. The VOE is reduced by 1.8%, 0.1%, 3.43%, 0.55%, 0.6%, and 3.17%, respectively; the RMSSSD is reduced by 0.9 mm, 0.1 mm, 1.08 mm, 0.93 mm, 0.1 mm, and 1.2 mm, respectively; and the MSSD is reduced by 10.1 mm, 3.2 mm, 8.6 mm, 12.1 mm, 6.7 mm, and 10.86 mm, respectively. Compared with [9, 11] and [31], the RVD decreased by 0.2%, 1.2%, and 0.1%, respectively. Compared with [9, 33, 34] and [32], the ASSD is reduced by 0.3 mm, 0.13 mm, 0.51 mm, and 0.49 mm, respectively, which further effectively demonstrates that the method in this paper can better segment the liver region.

Table 3 presents the results of the evaluation for segmentation accuracy of the proposed algorithm using five randomly selected CT data types on ISBI 2017 datasets.  Table 4 lists the comparison results of the segmentation errors of the method and [1] in the ISBI 2017. In the table, “—” indicates that the relevant value has not been calculated in the references. Compared with [1], the VOE is reduced by 0.14% and the ASSD is reduced by 0.67 mm. Its performance is slightly poorer than that of [1] in terms of the RVD and MSSD.

The hospital data includes 100 contrast-enhanced CT volumes.  Table 5 shows five groups of data randomly selected from the 100 CTs to verify the segmentation accuracy of the algorithm proposed in this paper. The quantitative results for these five data were 5.23 ± 0.6%, 2.3 ± 0.8%, 1.18 ± 0.4 mm, 2.25 ± 0.68 mm, and 17.2 ± 6.8 mm, respectively.

## 5. Discussion and Conclusion

In this paper, an efficient liver segmentation was proposed which was based on the Gabor dictionary of sparse image patches selected in prior boundaries from CT images. To solve the problem that the machine learning-based method needs a large number of training samples (which would affect the segmentation efficiency), this paper used the gold standard image and the target image to obtain the initial boundary of the liver and selected the test sample set within the neighborhood of the initial boundary, effectively reducing the number of samples. In the Gabor image of the training image, an image patch corresponding to the liver boundary was selected to construct an inquiry dictionary and two sets of inquiry dictionaries were used to obtain the corresponding sparse coefficients, effectively expressing information about the liver boundary by combining the inquiry dictionary and sparse coefficients. In addition, the reconstruction error of the test sample and the inquiry dictionary was optimized. The center of the image patch with the smallest reconstruction error was used as the liver boundary, and the segmentation model was completed and filled by applying the void-filling method to the liver surface, which ensured the smoothness and accuracy of the segmentation result.

The method for liver segmentation was validated with two popular public datasets and clinical datasets. In the MICCAI 2007 dataset, compared with the segmentation methods proposed in recent years, our method has improved in VOE, RMSSSD, and MSSD. On the ISBI 2017 dataset, the ASSD value of this method is 0.67 mm lower than that proposed by Qin et al. Our methods are competitive with previous methods in both accuracy and efficiency, and we validate the proposed method in clinical datasets. The results proved the validity of the Gabor information mentioned in this paper in establishing an inquiry dictionary. In addition, it can also be concluded from the experiment that the segmentation results after void filling were obviously more accurate than the results that did not undergo the void filling process. After void filling, the discontinuity and local overlap of the segmentation result was also repaired, which shows that the algorithm in this paper can realize the accurate segmentation of the liver in CT images.

However, since the method proposed in this paper mainly uses the registered and deformed liver model as the initial boundary of the target image and selects the image patch within the initial boundary as the test sample set, accurate liver boundary segmentation could not be achieved for large deformed regions that have not been registered accurately.

## Figures and Tables

**Figure 1:** Architecture of liver segmentation.

**Figure 2:** Registration flow chart.

**Figure 3:** Schematic diagram of the training set selection. In the figure, the left is the grayscale image with the “gold standard,” the middle is the schematic diagram of selecting image patches in corresponding Gabor images, and the right is a locally amplified graph.

**Figure 4:** Registration process and results: (a) the training image, (b) the gold standard image of the liver relative to (a), (c) the deformed version of registered image (a), (d) the gold standard image of liver relative to Figure (c), (e) the target image, where the points marked with (1)∼(5) in (a) and (e) are the selected marked points, and (f) the posture of the registered gold standard image of the liver in the target image.

**Figure 5:** Examples of registration results: (a)∼(f) how six sets of registration results are displayed in binary images.

**Figure 6:** Gabor dictionary.

**Figure 7:** Images of the image patch selection results of the dictionary in the slice. (a)∼(c) are 3 sets of liver data. The first column to the third column is the display effects of the training set on the cross section, sagittal plane, and coronal plane, respectively.

**Figure 8:** Results of the liver boundary point set obtained by the sparse dictionary method. (A1)∼(A3) and (B1)∼(B3) offer two sets of segmentation results, respectively. Columns 1–3 show the cross-sectional, sagittal, and coronal planes of the same data, respectively. (a1)∼(a3) are the locally amplified views corresponding to the green boxes in (A1)∼(A3), respectively.

**Figure 9:** Segmentation results. In the figure, the three columns are the coronal plane, cross section, and sagittal plane of liver segmentation results, respectively. The last three rows are partially enlarged views corresponding to the first three rows of images.

**Figure 10:** Segmentation results of five sets of liver data.

**Figure 11:** Three-dimensional display comparison diagram of the liver segmentation results.

**Table 1:** Quantitative evaluation of segmentation results on MICCAI 2007 datasets.

Data number	VOE (%)	RVD (%)	ASSD (mm)	RMSSSD (mm)	MSSD (mm)
1	4.54	0.7	0.65	0.71	9.16
2	4.9	2.58	1.03	1.89	16.91
3	4.16	1.24	0.42	0.97	6.33
4	4.78	1.67	0.82	1.4	12.8
5	5.28	2.02	1.26	1.71	18.42
Average	4.7 ± 0.4	1.6 ± 0.7	0.8 ± 0.3	1.3 ± 0.5	12.7 ± 5.1

**Table 2:** Comparative results with previous methods on MICCAI 2007 datasets.

Method	VOE (%)	RVD (%)	ASSD (mm)	RMSSSD (mm)	MSSD (mm)
Proposed method	4.7 ± 0.4	1.6 ± 0.7	0.8 ± 0.3	1.3 ± 0.5	12.7 ± 5.1
Ref. [11]	4.8 ± 0.7	1.8 ± 0.4	**0.8** **±** **0.1**	1.4 ± 0.4	15.9 ± 4.3
Ref. [9]	6.5 ± 0.6	2.8 ± 0.9	1.1 ± 0.3	2.2 ± 0.8	22.8 ± 7.6
Ref. [31]	8.13 ± 2.08	0.42 ± 3.64	1.31 ± 0.44	2.38 ± 0.68	21.35 ± 3.27
Ref. [32]	5.3 ± 2.1	1.7 ± 1.5	0.8 ± 0.5	1.4 ± 0.7	19.4 ± 5.3
Ref. [32]	7.87	1.31	1.29	2.50	23.56

The bold values indicate that reference [11] is slightly better than our proposed method in RVD values.

**Table 3:** Quantitative evaluation of segmentation results on hospital datasets.

Data number	VOE (%)	RVD (%)	ASSD (mm)	RMSSSD (mm)	MSSD (mm)
1	4.05	1.65	0.64	1.66	6.24
2	5.65	3.2	1.32	3.19	20.64
3	5.16	2.08	1.14	2.21	15.84
4	4.61	0.94	0.96	1.14	10.16
5	6.07	2.64	1.46	2.8	26.16
Average	5.1 ± 0.8	2.1 ± 0.9	1.1 ± 0.3	2.2 ± 0.8	15.8 ± 7.6

**Table 4:** Comparative results with previous methods on ISBI 2017 datasets.

Method	VOE (%)	RVD (%)	ASSD (mm)	RMSSSD (mm)	MSSD (mm)
Proposed method	5.1 ± 0.8	2.1 ± 0.9	1.1 ± 0.3	2.2 ± 0.8	15.8 ± 7.6
Ref. [1]	5.24 ± 0.69	1.97 ± 1.7	1.77 ± 0.49	—	13.03 ± 5.71

**Table 5:** Quantitative evaluation of segmentation results on hospital datasets.

Data number	VOE (%)	RVD (%)	ASSD (mm)	RMSSSD (mm)	MSSD (mm)
1	4.33	1.93	0.64	1.77	7.84
2	5.18	2.27	1.2	2.38	17.28
3	5.51	3.47	1.46	3.1	21.74
4	4.95	1.27	0.92	1.42	12.96
5	6.17	2.73	1.7	2.73	26.26
Average	5.23 ± 0.6	2.3 ± 0.8	1.18 ± 0.4	2.25 ± 0.68	17.2 ± 6.8

## Data Availability

The MICCAI 2007 dataset is available at https://www.sliver07.org/index.php. The ISBI2017 dataset is available at https://competitions.codalab.org/competitions/17094#le-arn_the_details.
